This article has been retracted.

# Polymorphisms in MicroRNA Genes Associated with Schizophrenia Susceptibility but Not with Effectiveness of MECT

**DOI:** 10.1155/2021/1959172

**Published:** 2021-12-13

**Authors:** Danwei Zhang, Huihua Li, Kaimo Ding, Zhen Zhang, Si Luo, Guohai Li

**Affiliations:** ^1^Department of Psychiatry, Zhenjiang Mental Health Center, Zhenjiang, Jiangsu Province, China; ^2^Department of Psychology, Zhenjiang Mental Health Center, Zhenjiang, Jiangsu Province, China

## Abstract

Schizophrenia (SCZ) is a common and complex psychiatric disease associated with hereditary and environmental risk factors. MicroRNAs (miRNAs or miRs) are small, noncoding RNA molecules that endogenously regulate gene expression. Single nucleotide polymorphisms (SNPs) in related miRNA genes are associated with susceptibility of the disorder. We wonder if the SNPs have influence on the effectiveness of modified electroconvulsive therapy (MECT) for SCZ. rs1625579 within miR-137, rs6577555 within miR-34, and rs2296616 within miR-107 were sequenced in 150 cases and 150 controls to check the potential association between the SNPs and SCZ. Our results showed that allele G in rs1625579 (*p* = 0.005, adjusted OR = 1.379, 95%CI = 1.108 − 1.634), allele A in rs6577555 (*p* = 0.014, adjusted OR = 1.246, 95%CI = 1.045 − 1.463), allele G in rs2296616 (*p* < 0.001, adjusted OR = 1.646, 95%CI = 1.374 − 1.879) are positively associated with the disorder risk. MECT courses did significantly decrease the level of the miRNAs, except for the variant of rs2296616 with the AA genotype. Schizophrenic phenotypes assessed by the positive and negative syndrome scale (PANSS) were improved after MECT, and there was no significant relevance observed between the effectiveness of MECT and the variants of these loci. Thus, our findings indicate that polymorphisms within the loci may be involved in the pathogenesis of SCZ, and MECT is effective and unbiased for patients harboring different genotypes of the loci.

## 1. Introduction

Schizophrenia (SCZ) is a common mental disorder manifested as psychosis, hallucinations, delusions, reduced expression of emotions, strange speeches, and a decreased capability to cognize reality, and about 0.7% of people are affected by SCZ in their lifetimes [1]. In 2013, there were around 23.6 million SCZ cases in the world [2]. Despite much progress in the investigation on SCZ, the precise cause of the psychiatric disease remains elusive. Lichtenstein et al. claimed that hereditary factors might play a major role in the occurrence of SCZ [3]. Recently, several studies showed that aberrant expressed microRNAs (miRNAs or miRs) observed in the serum [4] and post-mortem brain tissue [5, 6] of SCZ patients compared with that of normal controls, which provided clues that miRNA may be an important element in the pathogenesis of SCZ.

miRNAs are short and noncoding RNAs of 19–25 nucleotides which can interact with the 3′-untranslated region (UTR) of targeted mRNAs to negatively modulate the expression at the posttranscriptional level [7, 8], which is believed to regulate approximately 60% of encoding genes [9] and play a vital role in various biological processes [10]. In the studies on SCZ, miR-34 expression was found to be associated with the disease in peripheral blood mononuclear cells in a meta-analysis involving 330 patients and 202 healthy controls [11]; miR-107 was also significantly upregulated in the dorsolateral prefrontal cortex of SCZ patients [6]. Single nucleotide polymorphisms (SNPs) within miRNAs can result in abnormal expression or secondary structural changes of the products [12, 13]. Some genome-wide association studies (GWASs) have suggested that several SNPs within miRNAs are associated with SCZ susceptibility [14]. For example, miR-137 rs1625579 was identified as a risk locus for SCZ in a GWAS analysis performed by the Psychiatric Genomics Consortium (PGC) [15]. This SNP locus in miR-137 is on chromosome 1p21.3, which was found to be the strongest predictor of SCZ risk in the analysis [16]. Thus, it would be valuable to further study the roles of SNPs within miRNAs in SCZ. Herein, we will focus if there is an association between the effectiveness of modified electroconvulsive therapy (MECT) and the SNPs in related miRNAs.

MECT is an effective treatment to mood disorders and has been used in the field of psychiatry for seven decades [17]. Nowadays, MECT is used as an enhancement of antipsychotic treatment and to solve drug-resistant symptoms in SCZ [18]. According to the report by Ward et al., the majority of patients with SCZ who receive MECT improved [19], but there was a significant difference in the therapeutic effect among patients. Therefore, we hypothesize that the SNPs in related miRNAs may cause the difference in effectiveness of MECT in SCZ treatment.

In order to investigate the influence of miRNA polymorphisms on MECT, three SCZ-related miRNAs mentioned above were selected, and rs6577555 within miR-34, rs2296616 within miR-107, and rs1625579 within miR-137 were genotyped in a case-control study including 150 clinically diagnosed SCZ and 150 healthy individuals. Furthermore, association of the SNPs with the effectiveness of MECT was evaluated according to PANSS scores in the present study.

## 2. Materials and Methods

### 2.1. Participants

In the case-control study, 150 clinically confirmed SCZ patients (82 males and 68 females at age 40.24 ± 9.55 years) according to the Diagnostic and Statistical Manual of Mental Disorders, Fourth Edition (DSM-IV) were recruited at Zhen Jiang Mental Health Center, Zhen Jiang, China. 150 healthy controls (80 males and 70 females at age 41.03 ± 7.82 years) were recruited from the community. The controls were checking-up individuals without personal or familial neuropsychiatric disorder history or any drug addiction. All of the participants were Chinese Han descendants ethnically. This research was approved by the ethics committee of the Zhen Jiang Mental Health Center, and written informed consent was obtained from all the subjects.

### 2.2. SNP Genotyping

Genomic DNA was isolated from the peripheral blood using a blood genomic DNA extraction kit (TIANGEN, Beijing, China). The 3 SNPs were detected by a TaqMan genotyping discrimination assay, and an ABI Prism 7900 Sequence Detection System (Applied Biosystems, Foster City, CA, USA) was employed in the assay. The primers are listed in Table 1. For quality control, 5% were repeated for the genotyping assay, and the results were more than 99% concordant. The experiments were carried out according to the manufacturer's protocols.

### 2.3. qPCR Assay

Total RNA was extracted from the samples using a TRIzol reagent (Invitrogen, Carlsbad, CA, USA). RNA was then reverse transcribed by a TaqMan microRNA Reverse Transcription Kit (Applied Biosystems, Foster City, CA, USA). The quantitative results were normalized to the expression of U6. The relative expression of genes was calculated using the 2^-∆∆Ct^ method. The primers used were listed as follows: miR-137, 5′-GCGCGC TTATTGCTTAAGAATAC-3′ (forward) and 5′-GTGCAGGGTCCGAGGT-3′ (reverse); miR-34, 5′-TCTATTTGCCATCGT-CTA-3′ (forward) and 5′-CAGGCAGCTCATTTGGAC-3′ (reverse); miR-107, 5′-AGCAGCATTGTACAGGG-3′ (forward) and 5′-GTGCAGGGTCCGAGGT-3′ (reverse); and U6, 5′-GCTTCGGCAGCACATATACTAAAAT-3′ (forward) and 5′-CGCTTCACGA-ATTTGCGTGTCAT-3′ (reverse).

### 2.4. Modified Electroconvulsive Therapy

All SCZ patients underwent medication washout for at least 14 days before being engaged into this study. The patients received modified bifrontotemporal ECT using Thymatron DGx (Somatics LLC, Lake Bluff, IL, USA), a brief-pulse, constant-current apparatus at Zhen Jiang Mental Health Center, Zhen Jiang, China [20]. The first three MECT courses were administrated on continued days, the remaining courses of MECT were performed every other day, and it would have a break on weekends. MECT was continued up to twelve courses. Anesthesia was induced with succinylcholine (0.5–1 mg/kg) and diprivan (1.5–2 mg/kg).

### 2.5. PANSS

Symptom severity was assessed by the positive and negative syndrome scale (PANSS) that is composed of 33 items, rated from 1 to 7 scores each. All the items are arranged into a positive subscale, negative subscale, general psychopathology subscale, and additional subscale to reflect the severity of SCZ [21]. PANSS assessment was conducted twice before the first and after the last treatment.

### 2.6. Statistical Analysis

Genotype frequencies of the three loci in cases and controls were acquired by counting. The Hardy-Weinberg equilibrium (HWE) was verified for the two groups. The two-tailed estimation of significance was chosen to evaluate the difference in quantitative results, and Pearson's chi-square test was used for examination of the distribution of the allele or genotype between the two groups. Odds ratio (OR) and 95% confidence interval (95% CI) were used to estimate the association between the SNPs and SCZ susceptibility. All statistics were performed using SPSS software 18.0 (SPSS Inc., Chicago, IL, USA), and *p* < 0.05 was considered statistically significant.

## 3. Results

The demographic characteristics and clinical variables of the SCZ and control groups are shown in Table 2. No significant difference was observed in age, sex, and status of smoking and drinking between the two groups.

We first sequenced the 3 SNPs in the miRNAs (miR-34a rs6577555, miR-107 rs2296616, and miR-137 rs1625579) with minor allele frequency (MAF) > 5% (Table 1). The genotype and allele distributions within them between the case and control groups were recorded in Table 3. The *p* values of HWE in all SNPs were larger than 0.05 (*p* value = 0.053 for rs1625579; *p* value = 0.104 for rs6577555; *p* value = 0.08 for rs2296616), indicating that genotypes of the loci were conformed to HWE. Genotype TT, TG, and GG and allele T and G frequencies of rs1625579 within miR-137 in the two groups were 74.67%, 84.67%, 17.33%, 13.33%, and 8.0% and 2.0%, 83.33%, 91.33%, 16.67%, and 8.67%, respectively. Comparing with genotype TT of the locus, the frequency of genotype GG (*p* = 0.026, adjusted OR = 1.707, 95%CI = 1.073 − 2.060) was significantly increased in cases, but a difference of the heterozygous TG genotype was not significant between the two groups. A positive association was found between allele G of the locus and the risk of SCZ (*p* = 0.005, adjusted OR = 1.379, 95%CI = 1.108 − 1.634). The association was observed in both dominant (*p* = 0.045, adjusted OR = 1.329, 95%CI = 1.007 − 1.662) and recessive (*p* = 0.034, adjusted OR = 1.652, 95%CI = 1.043 − 1.986) models as well. Genotype CC, CA, and AA and allele C and A frequencies of rs6577555 within miR-34 in cases and controls were 54.00%, 60.67%, 26.00%, 31.33%, and 20% and 8%, 67.00%, 76.33%, 33.00%, and 23.67%, respectively. Comparing with genotype CC, the frequency of the homozygous AA genotype (*p* = 0.008, adjusted OR = 1.517, 95%CI = 1.121 − 1.882) was significantly increased on the locus in the case group. Allele A of rs6577555 was indicated as a significant factor positively associated with the risk of SCZ (*p* = 0.014, adjusted OR = 1.246, 95%CI = 1.045 − 1.463), which was verified in the recessive model (*p* = 0.005, adjusted OR = 1.536, 95%CI = 1.150 − 1.871). Genotype AA, AG, and GG and allele A and G frequencies of rs2296616 within miR-107 in cases and controls were 70.00%, 88.00%, 18.67%, 10.67%, and 11.33% and 1.33%, 79.33%, 93.33%, 20.67%, and 6.67%, respectively. In comparison with genotype AA of the locus, frequencies of genotypes AG (*p* = 0.028, adjusted OR = 1.436, 95%CI = 1.041 − 1.826) and GG (*p* < 0.001, adjusted OR = 2.020, 95%CI = 1.437 − 2.251) were significantly increased in cases, and a positive association was confirmed between allele G of the locus and the risk of SCZ (*p* < 0.001, adjusted OR = 1.646, 95%CI = 1.374 − 1.879). The relevance was also found in dominant (*p* < 0.001, adjusted OR = 1.612, 95%CI = 1.263 − 1.945) and recessive (*p* = 0.001, adjusted OR = 1.890, 95%CI = 1.353 − 2.100) models. These results indicated that the three polymorphisms of the loci are all relevant with the risk of SCZ occurrence.

The effectiveness of MECT was evaluated by PANSS. As shown in Table 4, all the total, positive symptom, negative symptom, and general symptom scores in the case group were decreased after MECT, indicating the improvements of the SCZ patients by MECT.

In Table 5, PANSS scores of the carrier with homozygous wild genotypes (TT genotype in rs1625579, CC genotype in rs6577555, and AA genotype in rs2296616) were generally lower than those with mutant homozygous or heterozygous genotypes. Moreover, the scores were all obviously decreased after MECT regardless of the genotypes. There was no association observed between the reduction of the PANSS scores and the SNPs. Thus, polymorphisms of the loci within these SCZ-related miRNAs had no significant influence on the effectiveness of MECT.

The levels of miR-137, miR-34, and miR-107 were significantly increased in the serum of SCZ patients compared with the controls (Table 6). The variants of miR-137 rs1625579 and miR-34 rs6577555 were decreased after MECT, including all genotypes (Tables 7–8). The AG/GG genotype of miR-107 rs2296616 decreased as well, but the AA genotype of the locus was not significantly changed after MECT (Table 9).

## 4. Discussion

Increasing evidence suggests that SCZ is a complex disease in which hereditary, environmental, psychological, and social factors are involved [22]. The psychiatric disease is resulted molecularly from malfunction of related protein encoding and noncoding genes that play a role in onset and development of the disorder. All of miR-137, miR-34, and miR-107 participate in the modulation of neuronal development and maturation [23–25] as well as the NMDAR signaling pathway and neurotransmission [25–27]. Genetic variants of these miRNAs may have a lower affinity to their targeted mRNAs and then contribute to the abnormal expression of encoding genes, ultimately triggering neuropsychiatric disorders including SCZ.

In the current study, we carried out a case-control study to investigate the association between the SNPs in related miRNAs and the disorder risk, and further to check the influence of the SNPs on the outcome of MECT for SCZ. Our results showed that allele G in locus rs1625579 was positively associated with the risk of SCZ, and the carrier with genotype TG/GG of the locus had higher PANSS scores compared to those with genotype TT in the case group, indicating that allele T of rs1625579 might be a protective factor for this disorder. These findings are consistent with the previous reports on this SNP in SCZ. Apart from the association with SCZ, miR-137 was also found to modulate neural stem cell proliferation and differentiation in fetal and adult mice [28]. Moreover, miR-137 overexpression inhibits dendritic morphogenesis, phenotypic maturation, and spine development both in the brain and primary cultured neurons [29]. Our data exhibited that MECT significantly decreased the level of miR-137 in the case group, which maybe a mechanism of the therapy to recover the neuron malformation and dysfunction in SCZ. Thus, miR-137 may be involved in the occurrence of SCZ by affecting neural connectivity, resulting in abnormal neural transmission.

The data on miR-34 rs6577555 showed allele A of the locus conferred a risk of SCZ onset according to the comparison between the control and case groups. The PANSS scores of patients harboring CA/AA genotypes were larger than those with the wild CC genotype. Overexpression of miR-34 in vitro significantly increased precursor proliferation and influenced morphology and function of developing neurons [30]. In the mature neuron, miR-34 overexpression decreases the levels of several synaptic proteins and receptor subunits but leads to a more efficient response to synaptic stimulus. However, the effects of miR-34 overexpression are just stage-specific in vivo [25]. miR-34 was found to be upregulated significantly in the blood sample of SCZ patients. The constant overexpression of miR-34 in SCZ may generate adverse influences on nervous function.

Polymorphism of rs2296616 within miR-107 was shown a significant association with susceptibility to SCZ in the current study. miR-107 is upregulated in dorsolateral prefrontal cortex from schizophrenic patients, which downregulates the expression of NMDAR subunit 3A; thus, it contributes to dysfunction of NMDAR signaling pathway, resulting in an increased SCZ risk [31]. This molecule is also highly enriched in pathways related with neural connectivity and synaptic plasticity, such as Wnt and MAPK signaling [32, 33]. The exact role of miR-107 in SCZ remains to be elucidated in further studies.

Apart from the genotype frequencies of these loci, we checked whether there was relevance between the variants and the effectiveness of MECT as well. The PANSS scores of patients were significantly decreased regardless of the genotypes of the loci, so we did not find any allele significantly result in resistance to MECT. The levels of most of the miRNA variants decreased after MECT, except for the AA genotype in miR-107 rs2296616. These results proved that MECT is a reliable and augmented treatment besides antipsychotic medications for SCZ patients.

In conclusion, the results of our case-control study provide convincing evidence that the polymorphisms of rs6577555, rs2296616, and rs1625579 are associated with SCZ risk. In addition, the outcome of MECT has no relevance with the variants of the loci. Further investigations on the functional consequences of these polymorphisms may help to elucidate more molecular mechanisms by which the genetic variants affect the schizophrenic phenotype.

## Figures and Tables

**Table 1:** SNPs in the miRNAs and primers in sequencing.

Gene	Location	Mutation	MAF	Sanger sequencing primers
miR-137	Chromosome	G>T	0.0667 (T)	F: 5′-ATG AGA ACA TCA TGG GGT CAC T-3′
rs1625579	1:98037378			R: 5′-GAT TCC AAA GGT CTC TAG TGT GC-3′
miR-34	Chromosome	C>A	0.2571 (A)	F: 5′-AAA GAG TCA GCA CTT CCC TGG-3′
rs6577555	1:9152228			R: 5′-GTT GGC GCT ACT TCA TTG CT-3′
miR-107	Chromosome	A>G	0.0667 (G)	F: 5′-GTG TTG CAC TGC CAA GAT GAT-3′
rs2296616	10:89593209			R: 5′-GGC TCC ATT GCT CGG ATG T-3′

MAF: minor allele frequency.

**Table 2:** Clinical characteristics of case and control groups in present study.

Characteristic	SZ (*n* = 150)	Control (*n* = 150)	*p* value
Age (years, mean ± SD)	40.24 ± 9.55	41.03 ± 7.82	0.43
Gender [*n* (%)]			
Male	82 (54.67%)	80 (53.33%)	0.82
Female	68 (45.33%)	70 (46.67%)	
Smoking [*n* (%)]			
Yes	52 (34.67%)	55 (36.67%)	0.72
No	98 (65.33%)	95 (63.33%)	
Drinking [*n* (%)]			
Yes	71 (47.33%)	68 (45.33%)	0.73
No	79 (52.67%)	82 (54.67%)	
Course of disease (months, mean ± SD)	40.5 ± 14.4		
PANSS scores (mean ± SD)			
Total	95.1 ± 14.9		
Positive symptom	26.9 ± 5.9		
Negative symptom	26.6 ± 7.6		
General symptom	41.5 ± 10.8		

**Table 3:** Genotype and allele distributions of rs1625579, rs6577555, and rs2296616 in cases and controls.

SNPs	SCZ (*n* = 150)	Control (*n* = 150)	*p* value of HWE	OR (95% CI)^∗^	*p* value^∗^	OR (95% CI)^#^	*p* value^#^
miR-137 rs1625579							
TT	112 (74.67%)	127 (84.67%)	0.053	1.000 (reference)		1.000 (reference)	
TG	26 (17.33%)	20 (13.33%)		1.474 (0.746-2.921)	0.23	1.206 (0.854-1.578)	0.299
GG	12 (8.00%)	3 (2.00%)		4.536 (1.152-20.814)	0.013	1.707 (1.073-2.060)	0.026
Dominant model				1.873 (1.014-3.474)	0.031	1.329 (1.007-1.662)	0.045
Recessive model				1.261 (1.089-19.458)	0.017	1.652 (1.043-1.986)	0.034
T	250 (83.33%)	274 (91.33%)		1.000 (reference)		1.000 (reference)	
G	50 (16.67%)	26 (8.67%)		2.108 (1.239-3.600)	0.003	1.379 (1.108-1.634)	0.005
miR-34 rs6577555							
CC	81 (54.00%)	91 (60.67%)	0.104	1.000 (reference)		1.000 (reference)	
CA	39 (26.00%)	47 (31.33%)		0.932 (0.536-1.620)	0.791	0.963 (0.705-1.282)	0.895
AA	30 (20.00%)	12 (8.00%)		2.809 (1.279-6.254)	0.005	1.517 (1.121-1.882)	0.008
Dominant model				1.314 (0.809-2.135)	0.243	1.145 (0.899-1.446)	0.293
Recessive model				2.875 (1.343-6.247)	0.003	1.536 (1.150-1.871)	0.005
C	201 (67.00%)	229 (76.33%)		1.000 (reference)		1.000 (reference)	
A	99 (33.00%)	71 (23.67%)		1.589 (1.092-2.312)	0.011	1.246 (1.045-1.463)	0.014
miR-107 rs2296616							
AA	105 (70.00%)	132 (88.00%)	0.08	1.000 (reference)		1.000 (reference)	
AG	28 (18.67%)	16 (10.67%)		2.200 (1.079-4.516)	0.018	1.436 (1.041-1.826)	0.028
GG	17 (11.33%)	2 (1.33%)		10.686 (2.296-68.554)	<0.001	2.020 (1.437-2.251)	<0.001
Dominant model				3.143 (1.654-6.018)	<0.001	1.612 (1.263-1.945)	<0.001
Recessive model				9.459 (2.045-60.437)	<0.001	1.890 (1.353-2.100)	0.001
A	238 (79.33%)	280 (93.33%)		1.000 (reference)		1.000 (reference)	
G	62 (20.67%)	20 (6.67%)		3.647 (2.081-6.443)	<0.001	1.646 (1.374-1.879)	<0.001

OR: odds ratio; 95% CI: 95% confidence interval. ^∗^Crude OR and 95% CI; ^#^OR and 95% CI were adjusted by age, gender and status of smoking and drinking.

**Table 4:** PANSS scores before and after MECT in the case group.

PANSS	Before MECT	After MECT	*t*
Total score	95.13 ± 14.91	54.50 ± 12.27	<0.001
Positive subscale	26.94 ± 5.91	14.87 ± 4.64	<0.001
Negative subscale	26.61 ± 7.58	18.05 ± 4.30	<0.001
General psychopathology subscale	41.51 ± 10.79	21.60 ± 7.90	<0.001

**Table 5:** Association between the SNP and PANSS scores in the case group before and after MECT.

	miR-137 rs1625579		miR-34 rs6577555		miR-107 rs2296616	
	TT (*n* = 112)	TG/GG (*n* = 38)	CC (*n* = 81)	CA/AA (*n* = 69)	AA (*n* = 105)	AG/GG (*n* = 45)
*PANSS before MECT*						
Total score	90.90 ± 13.66	107.58 ± 11.03	88.62 ± 13.36	102.77 ± 12.93	89.72 ± 12.76	107.73 ± 11.63
Positive subscale	25.67 ± 5.32	30.68 ± 6.05	25.42 ± 5.69	28.72 ± 5.70	25.45 ± 5.48	30.42 ± 5.45
Negative subscale	25.78 ± 7.67	29.08 ± 6.82	24.49 ± 6.86	29.10 ± 7.68	25.59 ± 7.66	29.00 ± 6.91
General subscale	39.46 ± 10.47	47.55 ± 9.46	38.58 ± 10.00	44.94 ± 10.73	38.59 ± 9.82	48.31 ± 9.92
*PANSS after MECT*						
Total score	52.42 ± 11.65	60.63 ± 12.11	51.26 ± 11.87	58.30 ± 11.69	51.67 ± 11.47	61.11 ± 11.60
Positive subscale	14.54 ± 4.63	15.84 ± 4.56	14.81 ± 4.99	14.93 ± 4.22	14.38 ± 4.52	16.00 ± 4.75
Negative subscale	17.70 ± 4.10	19.08 ± 4.76	17.11 ± 3.49	19.14 ± 4.89	17.48 ± 3.95	19.38 ± 4.81
General subscale	20.21 ± 7.60	25.68 ± 7.43	19.37 ± 7.47	24.22 ± 7.64	19.84 ± 7.27	25.71 ± 7.88

**Table 6:** Levels of the miRNAs in the case and control groups.

	miR-137	miR-34	miR-107
SCZ	2.61 ± 2.06	4.10 ± 2.81	1.58 ± 1.35
Controls	1.99 ± 1.56	3.21 ± 2.62	1.09 ± 0.79
*t*	2.939	2.837	3.837
*p*	0.004	0.005	<0.001

**Table 7:** The level of miR-137 rs1625579 before and after MECT.

miR-137 rs1625579	Before MECT	After MECT	*t*	*p*
TT (*n* = 112)	1.64 ± 0.63	1.18 ± 0.98	4.179	<0.001
TG/GG (*n* = 38)	5.53 ± 1.70	3.93 ± 1.23	4.700	<0.001
*t*	13.788	13.976		
*p*	<0.001	<0.001		

**Table 8:** The level of miR-34 rs6577555 before and after MECT.

miR-34 rs6577555	Before MECT	After MECT	*t*	*p*
CC (*n* = 81)	1.83 ± 0.62	1.51 ± 1.11	2.265	0.025
CA/AA (*n* = 69)	6.77 ± 1.64	4.93 ± 1.34	7.217	<0.001
*t*	23.624	17.097		
*p*	<0.001	<0.001		

**Table 9:** The level of miR-107 rs2296616 before and after MECT.

miR-107 rs2296616	Before MECT	After MECT	*t*	*p*
AA (*n* = 105)	1.01 ± 0.37	0.91 ± 0.41	1.855	0.065
AG/GG (*n* = 45)	3.16 ± 1.33	2.27 ± 0.84	3.795	<0.001
*t*	10.669	10.346		
*p*	<0.001	<0.001		

## Data Availability

The data used to support this study are available from the corresponding author upon request.
